The article "A review on surface modification of nanofibrous textiles for diverse applications: Focus on medical uses" was retracted in 2026. Reasons: unreliable results or conclusions; concerns about the citations.

# A review on surface modification of nanofibrous textiles for diverse applications: Focus on medical uses

**DOI:** 10.1016/j.heliyon.2025.e41863

**Published:** 2025-01-10

**Authors:** Rasool Shabanloo, Majid Montazer, Ali Farahani, Nesa Karimi

**Affiliations:** a Textile Engineering Department, School of Materials and Advanced Processes Engineering, Amirkabir University of Technology (Tehran Polytechnic), Tehran, Iran; b Department of Polymer Engineering and Color Technology, Amirkabir University of Technology, Tehran, Iran

**Keywords:** Electrospun nanofibers, Surface modifications, Biomedical applications, Physical modification, Chemical modification

## Abstract

Electrospun nanofibers with a high surface area are attractive materials for biomedical applications. They have potential use in scaffolds, drug delivery, bio face masks, wound dressings, and biosensors. Various surface modifications have been developed to improve their chemical and physical properties. These modifications include physical, chemical, biological, and nano-treatment approaches. The physical modification includes annealing, stretching, and plasma treatment. Chemical modification includes functionalization with chemical groups, while biological modification involves coating with proteins, enzymes, or antibodies. Nanotreatment approaches use nanomaterials to modify the surface of nanofibers. These modifications enhance the characteristics of the biomedical nanofibers, making them more effective and efficient for their intended applications. The review summarizes the latest research on electrospun nanofiber modification procedures, strategies, and utilities for various biomedical applications. It provides insights into the conditions and requirements of each modification approach and their effects on the properties of the nanofibers. Moreover, it emphasizes the importance of functionalizing nanofibers to meet the most important specific requirements and the potential of electrospun nanofibers in various biomedical applications.

## Highlights

• Emphasizes importance of functionalizing nanofibers for specific requirements.
• Surface modifications improve properties of nanofibers for biomedical applications.
• Physical, chemical, biological, and nanotreatment approaches available for nanfibrous modification.
• Insights into conditions and requirements of each approach.
• Potential use in scaffolds, drug delivery, wound dressings, biosensors, bio-facemask.

## 1 Introduction

Nanofibrous materials offer several advantages, including high surface area-to-volume ratio, porosity, and flexibility. These make them attractive candidates for medical applications, such as tissue engineering, drug delivery, wound healing, and medical implants [1]. Surface modification of nanofibers is an important technique for improving their properties and functionality, making them suitable for various applications, including biomedical applications.

The concept of “nanofiber surface modification” has been floated because, despite its simplicity, it is a complex process with no guarantee of success. Scientists have been widely working on modifying nanofibrous materials (Fig. 1). The surface of nanofibrous membranes is often modified through coating, deposition, and electrostatic attraction, among other approaches [2].

**Fig. 1:** Number of publications on modification of nanofibrous materials (Adapted from PubMed).

Electrospinning is one of the most common techniques for producing nanofibrous materials for wound healing. It allows for the nanofibers' production with controllable fiber diameter, porosity, and surface area, making them ideal for wound healing. The electrospinning technique facilitates the creation of interconnected networks composed of fibers with a nano-scale diameter, closely resembling the natural extracellular matrix structure [3]. This similarity enhances the standard cellular activities, including supporting cell attachment and promoting proliferation [4]. Electrospun wound dresses offer great compliance and flexibility with comfort once they are in place. Dressings made from biodegradable polymers through electrospinning may enhance patient comfort and adherence because they require fewer changes. Additionally, biodegradable electrospun wound dressings promote healing and accelerate cell growth due to their excellent compatibility with blood and tissues. The degradation rate of these scaffolds can be adjusted to the rate of tissue regeneration [5,6]. Surface modification of electrospun nanofibers can further improve their performance and properties, making them suitable for specific applications [7]. For instance, nanofibers in wound dressings have been widely studied due to their ability to mimic the extracellular matrix (ECM) of the human body [8]. Moreover, multifunctional wound dressings can reduce wound healing time and extend the dressing application [9,10].

Nanofiber surface modification can be achieved through various techniques, including physical, chemical, and biological approaches. The most commonly used method for surface modification of nanofibers is physical adsorption, which involves the adsorption of molecules onto the surface of the nanofibers [11]. This technique is simple, cost-effective, and can be used to modify the surface properties of nanofibers without altering their bulk properties. Other methods, such as chemical modification and biological functionalization, involve the covalent bonding of molecules to the surface of the nanofibers, resulting in more stable modifications [12]. These surface-modified nanofibers can be utilized in a wide range of applications.

One of the most promising applications of surface-modified nanofibers is developing bio-masks to prevent infectious diseases, such as COVID-19. Nanofibers in bio-masks can provide high filtration efficiency, breathability, and comfort. Nanofiber surface modification can further enhance bio-mask performance by adding functionalities such as antimicrobial activity and self-cleaning properties [13].

There is much interest in plasma treatment as a low-cost and green process. The electrospun polylactic acid nanofibers treated with gelatin may be more compatible with cartilage cells used for regeneration. The scaffolds were enriched with carboxylic groups using oxygen plasma and a coupling chemical to attach cationized gelatin (water-soluble carbodiimide). Compared to controls, the scaffolds improved chondrocyte viability, proliferation, and differentiation in rabbit joints [14].

The layer-by-layer (LBL) fabrication of electrospun nanofiber membranes using electrostatic attraction is becoming more preferred by researchers. Using negatively charged phosphotungstic acid, then positively charged polyethyleneimine (PEI) and silver nanoparticles (NPs) on electrospun nanofibrous produced a high photocatalytic performance [14]. Although loading functional materials such as metal oxides, NPs, and functional groups is straightforward, the endurance and stability of these materials are still tricky. Chemical grafting of nanofibers may effectively compensate for this defect. However, chemical grafting is possible to combine a specific functional group in a nanofiber. The adsorption or separation efficiency may be considerably improved using the composite electrospun nanofibrous in conjunction with the target active group [15]. In addition, chemical grafting of dopamine and graphene-based nanofibrous may produce antibacterial and hydrophilic characteristics [16]. Polylactic acid nanofibers were grafted with dopamine methacrylamide monomer-change graphene oxide (GO) through linked catechol and displayed excellent antibacterial efficacy against Gram-positive and negative bacteria [17]. Therefore, a comprehensive review is needed to cover recent developments and applications of nanofibrous and textile materials. This review will focus on the surface modification of nanofibrous materials for medical applications. The use of nanofibers in medical applications holds great promise due to their unique properties and the ability to modify their surface properties to suit specific applications. The development of surface modification techniques for nanofibers has further expanded their potential use in medical applications, allowing for enhanced biocompatibility, drug delivery, and pathogen filtration capabilities.

This review discusses various surface modification techniques such as physical, chemical, bio, and nano treatment and their effects on the properties of nanofibers. In addition, this review will cover the recent advances in surface modification techniques and their potential use in medical applications.

## 2 Electrospinning for the production of nanofibrous materials

Producing polymer solution filaments using electrostatic rather than mechanical forces can be unique [18]. As shown in Fig. 2, the polymer solution was first injected into a syringe with a desirable rate of injection, and then the proper droplets were created utilizing the appropriate feeding. An electric field is made after providing a required voltage on the anode and cathode, causing the traveling polymer jet to be ejected from the needle tip to the collector The collector rotates with appropriate speed when electric fields are more than a polymer solution surface tension.

**Fig. 2:** Common electrospinning setup.

Nanofibrous materials may be employed in various applications because of their remarkable characteristics, such as large specific surface area, proper porosity and pore size, and product thickness[[19], [20], [21], [22], [23]]. However, the limitations of electrospun nanofibers, such as hydrophobicity, lack of functional groups on their surface, and compatibility, restrict their potential in biomedical applications. Surface modification of electrospun nanofibers is a promising approach to address these limitations and enhance their bio-compatibility, mechanical properties, and functionality [24]. Different surface modification techniques including physical, chemical, biochemical, and nano treatment with bio-molecules were investigated to improve the properties of electrospun nanofibers for biomedical applications. (Fig. 3). These techniques can introduce functional groups on the surface of electrospun nanofibers, improve their hydrophilicity, and enhance their bio-compatibility [25]. For instance, surface modification with bio-molecules such as peptides or growth factors can promote cell adhesion, proliferation, and differentiation, making them suitable for tissue engineering and regenerative medicine applications. Thus, surface modification of electrospun nanofibers is an effective approach to enhance their properties for biomedical applications, and different techniques can be tailored depending on the specific application requirements [26].

**Fig. 3:** Different approaches for nanofiber modification.

## 3 Physical treatment on nanofibrous materials

### 3.1 Plasma treatment on nanofibers

Polymeric substrates have long been modified using plasma treatment to alter surface properties such as adhesion and wettability [[24], [25], [26], [27]]. Plasma treatment is more cost-effective and safer (no harmful solvent, less degradation of samples, and no chemical and toxic wastewater) than other methods of modification of textile materials [[28], [29], [30], [31]]. Nabil et al. have widely discussed the plasma treatment on cellulosic fabrics and their advantages and impacts on the environment. They mentioned plasma treatment as an efficient eco-friendly treatment that can be a promising substitute for chemical treatments [32]. The nanofibers' surface has been modified by plasma treatment (Fig. 4 and Table 1).

**Fig. 4:** Plasma treatment of nanofibers.

**Table 1:** Plasma treatment of different nanofibrous materials and their properties.

Plasma	Discharge gases	Nanofiber	Properties	Ref.
Radio frequency (RF)	O_2_, N_2,_ NH_3,_ HCOOH, H_2_O, CO_2_	Carbon	• Enhanced wettability • Incorporation of different functional groups	[33]
RF	Ar, O_2_	Carbon	• Increasing surface compatibility with the polymer surface	[34]
Atmospheric pressure glow discharge	Air	PCL	• Increase in wettability • Surface functionalization	[35]
RF	Ar, O_2_	Polycaprolactone (PCL)	• Enhanced cell adhesion and faster proliferation • Higher oxygen in the surface • Lower hydrophobicity	[36]
RF	O_2_	SnO_2_	• Higher specific surface area, porosity, absorbed oxygen, and response values • Low operating temperature • Higher selectivity to formaldehyde in the interfered gases of ethanol, ammonia, acetone, toluene, and methanol	[37]
RF	Ar/O_2_	Chitosan/poly (vinyl alcohol)	• Lower crystallinity and mechanical properties • Morphology alteration • Molecular backbone degradation and decomposition of polyene and carbonyl residues	[38]
RF	Ar, C_4_F_8_	Polyamide 6	• No changes in morphology • Better hydrophobicity Surface, and volume modification	[39]
DBD	O_2_	PVA/Aloe Vera	• Improved tensile strength, Young's modulus, and surface wettability	[40]
DBD	Ar, N_2_	PCL/chitosan	• Improved fiber wettability • Slight decrease in the surface roughness • Lower tensile strength	[41]
DBD	O_2_	PVA/Gelatin	• Improved tensile strength and Young modulus	[42]

Sunanda Roy et al. utilized radiofrequency oxygen plasma on cellulose nanofibers (CNFs) using glycerol (Gly) and glutaraldehyde (GA) to obtain antifogging properties. The radiofrequency oxygen plasma-treated sample depicts the most antifogging properties and wettability among the other samples. The tensile strength, tensile strain, young modulus, and toughness are the highest in 10 GA-8Gly-CNF film at 132 MPa, 4.2 %, 8 GPa, and 1660 kJ/m^3^, respectively [21]. Cold plasma can be used to increase protein interactions with cells [32]. Mozaffari et al. modified the gelatin nanofibers using argon and argon–oxygen plasma surface modification to prepare them for biomedical applications. The morphology of the nanofibers did not change notably. Untreated nanofibers were 300 ± 28 nm in diameter, whereas it was 294 ± 37 nm and 291 ± 45 nm for oxygen and oxygen-argon plasma treatment, respectively. An increase in wettability of the plasma-treated samples, confirmed with the water contact angle, due to the higher polar groups generated on the surface of the gelatin [34]. Cold plasma treatment can immobilize amine and oxygen polar functional groups to enhance cellular proliferation, adhesion, and viability on the nanofibrous mats [43,44].

### 3.2 UV treatment on nanofibers

Ultraviolet treatment (UV) is one of the most important, easy, and cost-effective ways of surface treatment of nanofibers since no chemicals and vacuum are needed for surface modification [45,46]. Tort et al. [47] considered the impacts of the UV on three-layer nanofiber within different times of UV exposure of 1, 2, and 3 h. The effects of exposure time on some essential properties, such as mechanical properties, wettability, morphology, and adhesion were investigated. The exposure time of 1h was insufficient to influence the microorganisms' internal structure to kill them. However, Duzyer et al. [48] sterilized the nanofiber after treatment with ethyl alcohol to decrease the microorganisms' density on the surface of the nanofibers. They showed an efficient exposure time for antimicrobial properties of 1 h. In addition, 1h and 2 h of sterilization had no significant impacts on mechanical properties, adhesion, and wettability, whereas 3 h of sterilization dropped the tensile strength from 2.76 to 2.05 MPa and contact angle from 39° to 30.5° with no significant effects on adhesion [47]. Other findings indicated that UV exposure for 2 and 3 h was adequate for sterilizing nanofiber wound dressings, however, 1 h proved insufficient to achieve complete sterilization. Although longer UV exposure time is more effective in reducing microorganisms, they may also impair the mechanical properties of the nanofibers [49]. Khosravi et al. worked on the activation of poly (ε-caprolactone) (PCL) by immobilizing silk-fibroin (SF) utilizing UV-ozone treatment. PCL nanofibers were modified using UV-ozone irradiation and acrylic acid. This approach immobilized SF via covalent bonding by functionalizing the surface of the nanofibers with active carboxylic groups. The surface modification approach increased the wettability of PCL nanofibers while introducing functional groups to the surface of the nanofibers. Furthermore, biological tests increased cell adhesion and proliferation [50]. Table 2 illustrates the Effect of UV treatment on different nanofibrous materials.

**Table 2:** Effect of UV treatment on nanofibrous materials.

Nanofiber	UV (nm)	Exposure time (h)	Properties after exposure	Ref
Poly (D, L-lactic-co-glycolic) acid (PLGA, 75:25) and poly(L-lactide-co-ε-caprolactone) [P(LLA-CL), 70:30]	254	1	• Significant degradation of nanofiber • Reduced molecular weight • Reduced tensile strength	[51]
Poly (lactic acid) (PLA)	254	1	• Unchanged morphology of nanofibers • Unchanged thermal and mechanical properties • Increased wettability	[52]
Linear polyethyleneimine (L-PEI)/polyvinylpyrrolidone (PVP)	(380–420)	0.5	• Improved solvent resistance, thermal stability, and mechanical properties • High cross-linking efficiency • Minimum toxic chemical residues	[53]
PVA/PAN	285	NA	• Controlled release • Improved chemical activity • Improved roughness	[54]

### 3.3 Microwave treatment on nanofibers

When microwaves ranging from 300 MHz to 300 GHz are utilized to treat materials, the energy may enter the dielectric substance directly, resulting in a quick and efficient heating process [55]. Microwave treatment has drawn a lot of attention in various applications. As mentioned in (Table 3) microwave irradiation was used to enhance the mechanical properties of chitosan/gelatin composite nanofibers as a polyelectrolyte complex (PEC).

**Table 3:** Microwave treatment of different nanofibrous materials and their properties.

Nanofiber	Microwave power	Exposure time (min)	Properties	Ref
Polyvinylpyrrolidone (PVP) /Titanium dioxide (TiO_2_)	0.75 kW	2–7	• Significant dispersion of Platinum (Pt) NPs without agglomeration • High electrochemical activity • Excellent electric catalytic activity • High stability of both catalytic activity and storage	[56]
Meta-aramid	12 kW/kg	6, 12, 18 (moist), 5,10,15 (wet) and 6 (dry)	• Higher thermal stability and crystallinity • More surface roughness • Inter-fiber cohesion • Reduction in CaCl_2_ Higher mechanical properties	[57]
Meta-aramid	12 kW/kg	3, 6, 9, 12 (wet) and 6 min (dry)	• Improved adhesion strength • Enhanced mechanical strength (tensile strength by 248.7 %) • Functional groups on nanofibers and increased wettability • Increasing the fiber alignment	[58]
Chitosan/gelatin	0.2, 0.4, and 0.6 kW	0.5,1,2	• Higher mechanical properties, crystallinity, swelling and antibacterial properties • More intermolecular interactions	[59]
Polyacrylonitrile (PAN)	0.1 kW	20–30	• Excellent and long-lasting antibacterial properties • Determined structure and uniform size of PAN-Ag^+^ micro/nanofibers	[60]
Cellulose di- and tri-acetate	1.4 kW	2–4	• Significant improvement in the morphology of nanofibers • Excellent degree of substitution and cellulose acetate yield	[61]

There is a lot of interest in using the microwave for organic synthesis [62], natural product extraction [63], and biomedical applications such as drug delivery control [64]. In materials processing, microwaves allow energy to be absorbed directly by the dielectric material, resulting in quick and uniform heating. The advantages of microwave treatment include its ability to penetrate rapidly and the ease of managing the treatment. For instance, Ning Cai et al. [65] created nanofibers using chitosan/gelatin and subjected them to microwave treatment at 600 W for 2 min. The microwave-treated nanofibers exhibited enhanced antibacterial effectiveness against both Gram-positive and Gram-negative bacteria, indicating their potential as a beneficial material for the treatment of infected wounds.

### 3.4 Gamma treatment on nanofibers

Many nanocomposites are gamma-irradiated to change their surface characteristics due to polymer excitation and chain scission/rupture or crosslinking [66,67].

Gamma-irradiation can improve the grafting effectiveness of biomaterial surfaces and the uniformity of bioactive peptides and protein molecules grafted on the surface, increasing wettability and cell survival [68,69]. Moreover, the addition of certain chemicals leads to chemical structure alterations [70]. Furthermore, some chemicals, such as heparin, can interact with and bind to proteins, and chemical or plasma treatments, and UV irradiation can result in increased toxicity and uneven surfaces [71]. To address these issues, gamma irradiation can be employed to enhance the grafting efficiency of bio-material surfaces and the uniformity of grafted bio-active molecules, including proteins and peptides, which can improve hydrophilicity and cell viability. Furthermore, uniform functionalization of the surface leads to controlled drug delivery [72,73]. The dosage of gamma irradiation of 15 KGy, on polystyrene/carbon nanotube (CNT) electrospun membranes depicted high hydrophobicity, antibacterial effect, and superior mechanical properties [74]. Polystyrene (PS) was filled with hexagonal boron nitride (hBN) and cobalt oxide (CO_3_O_4_) nanomaterials to make efficient and robust oil absorption. Utilizing these nanomaterials increased the interfacial contacts between the filler and polymer, improving tensile strength. Surface roughness was enhanced using gamma irradiation on the hydrophobic films (Fig. 5(a–f)). Increasing surface roughness was proved to be efficiently effective on hydrophobicity due to expanding the water contact angle from 140° ± 1 for neat PS fiber to 152° ± 2 for gamma-irradiated PS nanocomposite fibers. The superhydrophobicity made them a good candidate for oil separation even at higher temperatures [75]. Jin-Oh Jeong et al. used electrospinning to make the PCL nanofibers, and gamma irradiation was used to modify the hydrophilicity by grafting 2-aminoethyl methacrylate (AEMA). Heparin was introduced via the EDC/NHS reaction. The gamma-irradiation was applied to regulate the BMP-2 release from heparin that adsorbed using AEMA-grafted PCL scaffolds which proved to be a good candidate for designing biomimetic scaffolds [76]. Table 4 gives some additional data on the gamma treatment of different nanofibrous materials.

**Fig. 5:** **SEM images before gamma irradiation for (a) pure PS, (b) PS/Co-O, (c) PS/hBCo-O; and after gamma irradiation for (d) pure PS, (e) PS/Co-O; and (f) PS/hBCo-O fibers (Reproduced with permission of** [75]).

**Table 4:** Gamma treatment on different nanofibrous materials and their properties.

Polymer	Irradiation (kGy)	Effect on substrate	Application	Ref
Polystyrene	13	• More surface roughness • Super hydrophobicity	• Oil absorption	[75]
PCL	25	• Increase initial cell viability • Controlled cell growth	• Tissue engineering	[76]
Chitosan/polyvinyl alcohol (PVA)	50–200	• Decreasing tensile strength • Strong intermolecular hydrogen bonds	–	[77]
PCL	30.8	• Lower degradation rate • Higher mechanical yield stress • Significant increase in M_w_ and decrease in M_n_	• Scaffolds	[78]
Poly (L-lactide) (PLLA)	5, 10, and 25	• Increasing thermal stability and tensile properties • Excellent enzymatic degradation • Efficient crosslinking networks	• Tissue engineering • Biomedical • Appropriate base for cell growth	[79]
PLA/PANI	25	• Stronger interfacial interactions • Improved wettability, tensile strength, electrical and conductivity	• Biomedical • Tissue engineering	[80]
PCL	25	• The improved proliferation of fibroblast cells	• Wound dressing •Wound care	[81]

### 3.5 Laser treatment on nanofibers

Having control over the surface properties of polymeric substrates is of high significance. Laser treatment is one of the most critical and practical methods, offering a flexible approach [82,83]. Lingna He et al. modified the wettability of electrospun poly (ε-caprolactone) scaffolds utilizing an ultrashort pulse laser in different conditions. The use of femtosecond laser ablation to control the hydrophilicity of the scaffolds was examined as a versatile and straightforward approach. Three other air, O_2_, and CF_4_ gasses and different laser powers were analyzed, and several assessments were done on nanofibrous scaffolds. The increase in laser power from 1 to 8 mW decreased the water contact angle from 132 ± 2° to 116° for treatment in CF_4_. The wettability of samples treated in the air was lower than the treated in CF_4_. However, the rate of decrease was much higher for in-air treatment [84]. In another study, the surface of molybdenum disulfide (MoS_2_)-modified polyamide (PA6) electrospun nanofibers was investigated after altering the femtosecond laser pulse energy and scanning speed. EDX was performed to ensure the distribution of Mo and S elements on nanofibrous mats showing the appropriate distribution of Mo and S elements. The hydrophilicity of the nanofibrous membranes was enhanced over time and after about 15 s. All samples showed complete wetting behavior. Moreover, the threshold energy for removing material was measured to be 1.8 nJ [85]. Laser treatment can have a remarkable impact on surface topography resulting in the wettability of PLA nanofibers. These surface-modified nanofibers can then be used in cell attachment and growth, storage, and release of nutrients. Table 5 shows the different laser treatments on PLA nanofibers and their responses to water contact angles. Apart from laser parameters, total wettability changed from hydrophobic to hydrophilic [86].

**Table 5:** **Effect of laser treatment on the wettability of PLA nanofibers (reproduced with permission of** [86]**)**.

Lase parameters	SEM Image		Contact angle
Reference, without Laser treatment	Before laser treatment		
Q = 50 nJ dL = 20 μm dP = 25 μm	After laser treatment		
Q = 40 nJ dL = 20 μm dP = 25 μm			
Q = 47 nJ dL = 30 μm dP = 37.5 μm			

### 3.6 Ultrasound treatment on nanofibers

Vibrations having a frequency exceeding 17 kHz are known as ultrasonic (US) waves. The ultrasound effect is caused by acoustic cavitation in a liquid medium, which causes bubbles to develop, swell, and then violently collapse in less than a microsecond, releasing tremendous heat and generating short-lived hot spots. In addition, US can be used for many purposes, such as cleaning textiles such as needles of knitting machines, dispersion of dyes and preparing the bathe used for pretreatments at low temperatures, improving dye diffusion, and synthesis and deposition of nanomaterials on textile substrates [87]. Many studies use the US to enhance the surface of nanofibrous materials or create a new feature on nanofibers. For instance, Jianhua Ye et al. produced polyurethane (PU) nanofibers through electrospinning, immersed them into the cellulose nanofibrils (CNF), and sonicated them to assist in absorbing the CNF particles. A significant enhancement was reported in the mechanical properties and wettability of the fabricated CNF-absorbed PU scaffolds. Furthermore, treated scaffolds showed improved cell attachment compared to non-treated PU [88]. In another study, chitin nanofibers were produced and modified through esterification with maleic anhydride and ultrasound. The esterification enhanced the decomposition of chitin nanofibers during the ultrasound process. Moreover, increasing power and treatment time resulted in finer nanofibers and higher uniformity. However, ultrasound treatment did not remarkably affect the acetylation degree, whereas the degree of crystallinity increased with more ultrasound power and prolonged treatment time [89].

Physical surface modifications were widely used for nanofibrous materials due to their outstanding properties such as simplicity, environmentally friendly procedures, applying different functional properties such as hydrophilicity and hydrophobicity, antibacterial and antifungal, and improved mechanical properties without altering the bulk of the substrates or damaging the surface [90,91]. To affect surface functionality by modifying the chemical structure of the surface, plasma treatment has been widely used. It has been proven to enhance surface functionality in an environmentally friendly manner, which aligns with the ultrasound modification of nanofibrous materials [92]. Plasma treatment and UV treatment are cost-effective and safe (no dangerous solvent, less degradation of specimens, and no chemical and hazardous effluent) for modifying nanofibrous materials. Plasma treatment is the fastest method among all physical and chemical methods lasting from a few seconds to a few minutes [93]. This method produces different functional groups, such as amine, hydroxyl, and carboxyl, on nanofibers promoting biocompatibility, cellular proliferation, adhesion, and viability on the nanofibrous mats making them proper candidates for biomedical applications.

Using microwaves ranging from 300 MHz to 300 GHz on nanofiber may be very effective since the radiation can penetrate the surface directly and deeply to introduce available bioactive functional groups. As a result, biomolecule interactions with cells will be promoted using microwave-treated nanofibers [94]. Gamma irradiation proved to be another effective method for surface modification of nanofibrous materials. Numerous composite materials are gamma irradiated to modify their surface features because electromagnetic gamma rays stimulate a polymer and trigger chain scission/rupture or cross-linking [95]. Like UV treatment, gamma-irradiation may increase the ability of biomaterial surfaces in grafting and the homogeneity of transplanted bioactive protein molecules and peptides, enhancing wettability and cell interactions.

On the other hand, TiO_2_ NPs can improve photocatalytic properties. In some cases, two physical modifications can be applied simultaneously to activate the surface [96]. Several physical surface modifications can be scaled up for industrial applications without chemical-associated waste compared with wet chemical modifications.

In summary, modifying the surface of nanofibrous textiles with various physical treatments offers a variety of benefits and difficulties, each with unique characteristics that address certain medicinal uses. For instance, plasma treatment adds functional groups without altering the bulk characteristics of nanofibers to increase surface energy. However, consistency of alteration is difficult and necessitates exact control over process variables. Furthermore, UV treatment is a simple and affordable method to alter the surface of nanofibers, enhancing properties such as hydrophilicity and biocompatibility. The primary drawback is the possible deterioration of nanofibers due to UV rays, which might reduce the mechanical strength. Properties such as wettability and adhesion can be improved quickly and effectively by microwave treatment. Despite its benefits, if not well regulated, the process may cause considerable harm to the nanofibers due to uneven heating. Laser treatment improves characteristics such as surface roughness and functionalization by precisely and locally altering the surface. However, the primary challenge is the expensive and complicated equipment needed, along with the possible heat damage to the nanofibers. Nanofiber surfaces may be cleaned and functionalized using ultrasound treatment, which improves surface area and porosity. However, the process may cause mechanical damage to the nanofibers if not properly managed. The performance of nanofibres for medical applications may be greatly enhanced by the careful selection and optimized physical treatment, even if each has its benefits and disadvantages. Future studies should concentrate on creating more economical and effective ways to modify the surface as required while preserving the nanofibers structural and functional integrity.

## 4 Chemical treatments of nanofibrous materials

### 4.1 Chemical oxidation of nanofibrous materials

Chemical oxidation is a surface modification technique that has gained significant attention in the biomedical field due to its ability to enhance the surface properties of nanofibers [97]. The method involves the treatment of nanofibers with a strong oxidizing agent, such as sodium hypochlorite or hydrogen peroxide, which results in the formation of hydrophilic functional groups on the surface of the nanofibers [98]. These functional groups, such as carboxylic acid and hydroxyl groups, improve the hydrophilicity and biocompatibility of the nanofibers, making them more suitable for biomedical applications [99]. Moreover, introducing these functional groups can also facilitate the immobilization of biomolecules on the surface of the nanofibers, which can enhance their bioactivity and functionality. Chemical oxidation can be applied to various nanofibers, including synthetic and natural polymers, to improve their properties for wound healing, drug delivery, and tissue engineering applications. However, optimizing the chemical oxidation parameters, such as the concentration of the oxidizing agent and the duration of the treatment, is critical to achieving the desired surface properties without compromising the structural integrity and properties of the nanofibers [100].

For example, chemical oxidation has been used to modify the surface of PLGA nanofibers with carboxylic acid groups, facilitating the immobilization of chitosan and heparin to create a surface with enhanced anticoagulant properties [101].

It is important to carefully optimize the chemical oxidation parameters, such as the concentration of the oxidizing agent and the duration of the treatment, to achieve the desired surface properties without compromising the structural integrity and properties of the nanofibers. Furthermore, selecting the appropriate oxidizing agent is also critical, as different agents may produce other functional groups on the surface of the nanofibers.

### 4.2 Chemical grafting of nanofibrous materials

Chemical grafting is a technique that involves attaching functional molecules or polymers onto the surface of nanofibers to improve their properties for bio-medical applications [102]. The process consists of creating functional groups on the surface of the nanofibers and then attaching the desired molecules or polymers through chemical reactions such as esterification, amidation, or click chemistry [103]. Chemical grafting allows for precise control over the surface properties of the nanofibers, such as hydrophilicity, surface charge, and bio-compatibility. Furthermore, this technique can introduce a wide range of functional groups or bio-molecules onto the surface of nanofibers, such as peptides [102], antibodies [104], and enzymes [105], to impart specific biological functions.

Chemical grafting has been applied to various nanofiber materials, including synthetic and natural polymers such as polyethylene terephthalate (PET) [106], PCL [107], and cellulose [108]. For example, a study has reported the successful grafting of hyaluronic acid onto the surface of PCL nanofibers using a carbodiimide coupling agent. The resulting nanofibers showed better cell adhesion and proliferation, and improved mechanical properties compared to unmodified PCL nanofibers [109].

Although chemical grafting is a significant method for surface modification of nanofibers, there are several challenges and limitations. For instance, attaining a consistent grafting density across the surface of nanofibers can be challenging. Inconsistencies in grafting density can result in uneven properties and performance of the nanofibers. Consequently, managing the grafting density to guarantee uniform functionalization and prevent defects is essential [110]. In addition, chemical grafting methods, particularly those using strong oxidizing agents or requiring high temperatures, can compromise the structural integrity of nanofibers, resulting in diminished mechanical properties and functionality. Studies indicate that fine-tuning reaction parameters, including the coupling agent's concentration and the reaction's duration, is essential for preserving the structural integrity of nanofibers [111]. Moreover, scaling up the chemical grafting process while ensuring reproducibility is difficult. Changes in reaction conditions can result in inconsistencies from one batch to another. Consequently, it is crucial to standardize protocols to guarantee reproducibility [112]. Applying harmful chemicals and solvents during grafting raises significant environmental and safety issues. It is critical to create more sustainable and safer methods for grafting. Recent research has concentrated on creating environmentally friendly grafting techniques that reduce the reliance on dangerous chemicals [113]. Thus, careful optimization of the chemical grafting parameters is necessary to avoid damaging the structural integrity of the nanofibers or compromising their properties. The concentration of the coupling agent, reaction time, and temperature are important factors that must be carefully controlled to achieve the desired grafting density and functionalization [114,115]. A schematic of the chemical grafting is shown in Fig. 6.

**Fig. 6:** Chemical grafting on nanofiber functional groups.

### 4.3 Hydrolysis/aminolysis of nanofibrous materials

Hydrolysis or aminolysis of nanofibers is one of the most renowned ways of modification used for surface modification of nanofibrous materials to introduce functional amine, hydroxyl, and carboxyl groups (Fig. 7).

**Fig. 7:** Hydrolysis/aminolysis of nanofiber.

For instance, electrospinning produced PCL nanofibers to construct wound dressings with high medical and mechanical properties. The alkali hydrolysis was then used to ensure the improvement of attaching antibacterial agents. One of the most prominent antimicrobial peptides, pexiganan, was utilized to modify the antibacterial properties of PCL nanofibers. Efficient antibacterial properties improvement was reported against Gram-positive and negative bacteria.

Moreover, modified electrospun decreased the cytotoxicity and cell viability depending on the amount of pexiganan grafted to the nanofibers [116]. In another study, CNFs with a diameter of about 45 nm. were considered by utilizing acid hydrolysis, alkali treatment, and bleaching to remove the impurities and improve thermal properties [117]. The other study investigated the CNFs produced from bleached kenaf fibers after treating supercritical carbon dioxide (SC-CO_2_). Alippilakkotte et al. [118] improved the compatibility of electrospun poly (lactic acid) (PLA) nanofibers with biological conditions. Alkali hydrolysis first activated PLA films to add carboxyl groups to the surface and then covalently grafted with gelatin utilizing a coupling agent. Biological tests illustrated that hydrolyzed gelatin-grafted nanofibers were compatible with a detrimental impact on fibroblast cells.

Aminolysis is a well-known method for introducing an amine group to the surface of a wide variety of polymers to introduce a unique feature on the surface of nanofibrous materials. Razmshoar et al. used the second generation of poly amido amine dendrimer (PAMAM-G2) to aminolyze PCL ester bonds. The effects of different ratios of PAMAM-G2 and other mixing times were investigated. Moreover, dendrimers in the electrospinning solution enhanced the power of modified electrospun nanofibers against breast cancer cells (MCF-7). Furthermore, the presence of NH_2_ and OH groups as a result of the aminolysis reaction improved the wettability of PCL nanofibers, as confirmed by the contact angle values [119]. In a study, ethylenediamine with amine functional groups was used to modify the surface of films and electrospun aliphatic polyesters of PLLA, poly(lactide-co-caprolactone) (PLCL), and PCL. The treatment time directly affected the number of free amine groups, and its efficiency was greater on films than on the nanofibers. Generally, aminolysis of the nanofibers and the films led to more hydrophilicity, and the contact angles depended on the type of the polymer. It is argued that the lower efficiency of the aminolysis for nanofibers is due to the high crystallinity of nanofibers shells and the strong skin of the nanofibers inhibited the aminolysis reaction [120]. Ganjalinia and coworkers used the second generation of polypropylene imine dendrimer as an aminolysis agent to modify the PLLA surface. Different parameters were considered to study their effect on scaffolds' mechanical properties, morphology, and host-guest properties without pretreatment. The hydrophilicity of scaffolds enhanced After modification.

Furthermore, pH values indicated that PLLA biodegradation increased the acidic rate by secreting lactic acid for four weeks of treatment, causing significant immune cell infusion and inflammation in the medium. However, the PLLA/G2 scaffolds considerably lowered and stabilized the acidic rate by aminolysis response [121]. Shabanloo et al. utilized amine-terminated dendrimer and quaternary ammonium Gemini surfactant to modify the PLLA. The quaternary ammonium gemini surfactant and dendritic polymer successfully aminolyzed the PLLA and introduced amine end groups to the polymer chain. These functional groups increased the wettability, cell viability, adhesion, and mechanical and antibacterial properties [122].

Chemical surface modification is another method to modify the surface of the nanofibrous materials. The chemical surface modification may improve the hydrophilicity of the surface even deeper layer due to altering the chemical reactions, which can change the molecules. Chemical surface modification leads to permanent modifications as opposed to some physical treatments. After modifications, the surface alters permanently due to the formation of stable covalent bonding between the nanofiber surface and other desired molecules or functional groups. This can be related to the external functional groups exposed to different chemical stimuli [123]. An advantage of this method can be preparing bio-active sites for attaching and growing favorable cells. However, a disadvantage may be uncontrolled chemical functionalization that can alter the bulk characteristics of the nanofibers [124]. To prevent unfavorable reactions that can decrease the mechanical properties or even destroy the nanofibers, parameters of reactions such as reaction time, temperature, pH, processes, and concentration of reactors should be controlled. Another merit of this method is the reaction time, which can be much shorter than physical surface modification. Therefore, chemical treatment can be a proper time-saving method.

### 4.4 Nano surface modification of nanofibrous material

Nano treatments can be done by various methods, such as using nanostructure materials, nanolayer coatings, and introducing nanoroughnesses on the surface [125]. For instance, coating polyamide nanofibers with lipophilic and hydrophobic PDMS and ZnO NPs resulted in UV resistance and efficient oil separation from the water [126]. Nano-modification processes are performed on many nanofibers to improve or create special functions on their surfaces. For instance, silver NPs develop an antibacterial PAN-based thermally stabilized substrate. Silver-modified nanofibrous membrane showed notable antibacterial activity against *E. coli* and *S. aureus* bacteria [127]. Another type of nanomodification is nanolayer (also known as nanocoating), defined as the creation of one or more layers on a nanofibrous substrate surface with a thickness in the nano range. Obaid et al. [128] produced an electrospun nanofibrous membrane (ENM) which was then modified using two steps of coating with a metal-phenolic network (MPN) to use in the separation of water and oil. In another study, the functionalized multiwall carbon nanotubes (F-MWCNTs) loaded on PCL were introduced as a stiffener tensile strength optimizer, and surface roughness controller [129]. The surface of nanofibrous materials can be modified with NPs, significantly affecting different properties such as mechanical properties, wettability, and biological activities. NPs will improve the surface area and electron transmission at room temperature without much energy, making the modified nanofibers a promising candidate for biomedical applications. In addition, NPs with small sizes are appropriate compounds, used in imaging tools for in vivo imaging applications due to their photostability, narrow emission range, and extended excitation wavelength compared with biomaterials [130]. Several studies investigated the surface modification of nanofibers with NPs. For instance, Modifying the surface of nanofibers with silver NPs greatly boosts their antibacterial effectiveness. This alteration enhances biocompatibility and facilitates cell adhesion, rendering these nanofibers appropriate for applications in wound healing [131]. In addition, modifying nanofibers with gold NPs increases their ability to load drugs and facilitates controlled release. This method is especially beneficial for targeted drug delivery systems, leading to better therapeutic results [132]. Moreover, integrating hydroxyapatite NPs into nanofibers improves their mechanical strength and osteoconductive properties. This adjustment is essential for creating scaffolds in bone tissue engineering, facilitating improved integration with natural bone [133]. A study explored the use of electrospray for modifying the surface of cellulose tissues with chitin nanofibrils. Various solvent systems were used to produce a biobased and skin-friendly product. Then, the surface of the cellulose tissues was evenly coated with electrospray chitin nanofibrils. The biological assessment indicated that all treated samples were appropriate for applications on the skin [134]. Likewise, electrospraying of chitin onto nanofibers, produced by electrospinning of copolymer of poly(ethylene oxide terephthalate) and poly(butylene terephthalate) (PEOT/PBT) that contains CN/polyethylene glycol (PEG) as a pre-composite demonstrated notable antibacterial properties [135].

To conclude, chemical surface modification has its advantages and drawbacks. Hydrophilicity and biocompatibility can be enhanced through the chemical oxidation of nanofibrous materials by the functional groups on their surface. However, it can also lead to degradation of the nanofiber structure and requires careful control of reaction conditions to avoid excessive oxidation. On the other hand, chemical grafting provides a versatile approach to introduce a wide variety of functional groups onto the nanofiber surface, enhancing properties such as antimicrobial activity and cell adhesion. The main challenge lies in achieving uniform grafting and maintaining the mechanical integrity of the nanofibers during the process. In addition, hydrolysis/aminolysis treatments are effective for introducing amino and hydroxyl groups, which can significantly improve the interaction between the nanofibers and biological tissues. Despite their effectiveness, these methods can sometimes result in partial degradation of the nanofibers and require precise control to avoid compromising the material structural integrity. Lastly, Nano surface modification techniques, such as the deposition of nanoparticles, offer the potential to impart multifunctional properties, including enhanced mechanical strength, higher reactivity, and antimicrobial activity. The primary disadvantage is the complexity and cost associated with these techniques, as well as the potential for nanoparticle agglomeration, which can affect the uniformity of the surface modification.

### 4.5 Surface biomodification of nanofibrous material

Enzymes have been proven to be effective, non-toxic, and environmentally friendly bioprocess chemicals [136]. Fig. 8 depicts the most important enzymes and their applications in modifying nanofibrous materials.

**Fig. 8:** Most important enzymes and their applications for different nanofiber modification.

There are natural biocatalysts with high specificity and efficiency that catalyze various processes with excellent selectivity [137]. Because of their nature and versatility, they are a worthy option for satisfactory chemical manufacture, biosensing creation, protein breakdown and analysis, biofiltration, and the food supply [138,139]. Recently, the immobilizing enzyme has been an exciting topic that has drawn much attention to coating the enzymes through the electrospinning method. Physical or chemical processes can be utilized to immobilize enzymes. Physical immobilization of enzymes includes adsorption, entrapment, or encapsulation. In the physical adsorption, enzymes weakly bonded to the support by the Van Der Waals force. Therefore, although physical adsorption is one of the simplest methods to immobilize enzymes, they can be easily separated [140]. Siqueira et al. [141] synthesized PLA/chitosan nanofibers and used an adsorption technique to immobilize lipase. The nanofibers retained a significant level of enzyme activity for up to 120 % compared to free lipase. However, the lipase-immobilized fibers could only be reprocessed for five cycles which can be related to poor bond strength between support and enzyme in the adsorption method.

On the other hand, the encapsulation method can be utilized as an effective way of preventing enzyme disruption and increasing enzyme loading capacity. This is a simple method of using several enzymes in nanofibers [142]. Xia et al. worked on the encapsulation of enzymes in nanofibers utilizing the co-electrospinning method. In addition, there are cases where enzymes and polymers co-electrospun simultaneously to make enzyme-encapsulated bioactive nanofibers [143]. Regarding chemical methods, chemical bonding has been widely investigated as an effective tool for immobilizing enzymes on specific sites and preventing enzymes from being separated [144]. Both the enzyme and the chitosan-based nanofibers may react through cross-linking. This form of cross-linking allows each enzyme to be attached via covalent bonds. Cross-linking can limit enzyme leakage from support when comparing physisorption to chemisorption Physical and chemical adsorptions normally depend on acid pH in which protonation of amino groups of chitosan starts. Hence, this method can also be used for stable enzymes at pH 7–8.5. Although cross-linking has maximum results in modifying linkages between enzymes and chitosan nanofibers, these modifications can also cause changes in the enzyme conformation, lowering the enzyme catalytic activity [145].

Lee et al. [146] immobilized α-chymotrypsin on pristine silk fibroin (SF) nanofibers. The maximum storage stability was demonstrated by α-chymotrypsin on SF nanofibers with a diameter of 205 nm, which maintained more than 90 % of its original activity after 24 h of treatment. Nanofibers with a 320 nm diameter possessed over 45 % of the primary activity, with the maximum stability in ethanol. In another study, lipase was immobilized on poly (acrylonitrile-co maleic acid) nanofibers covalently by a straightforward method. The activity retention of the immobilized nanofibers was 37.6 %, and the amount of lipase loaded on nanofibers was 21.2 mg/g fibers. The loading and behavior of the enzyme can be flexibly customized considering the types of nanofibers, immobilization strategies, and treatment procedures for the supports. However, it is impossible to prevent the decline in enzymatic activity. Jahanfar and his coworkers modified the PVA/PAN nanofibers using dielectric barrier discharge plasma (DBD) to immobilize glucose oxidase (GOx). Different exposure times were investigated, and 6 min was selected as the optimum time. Intriguing results showed that plasma-treated samples had higher enzyme activity than untreated samples. Moreover, good enzyme retention and stability were reported for modified samples [147].

Cellulase is an enzyme that helps catalyze the hydrolysis of 1,4-D-glucosidic bonds in cellulose, forming the major component of plant cell walls. Cellulases and related enzymes are also in demand due to the increased interest in turning lignocellulosic biomass into fermentable sugars‏ [148]. Cellulase has been widely used in biomedical applications along with CNFs to attain controllable biodegradation of CNFs. Tamo et al. [149] loaded cellulase, alginate microparticles CNF as a carrier for releasing the enzyme and biodegradation of CNFs. Because of the high surface area of the alginate microparticles, releasing the encapsulated cellulase was effectively done in a controlled manner leading to appropriate hydrolysis of CNFs. After a day, the encapsulated enzyme activity stabilized at about 60 % and remained stable for three weeks.

Similarly, cellulase was encapsulated in chitosan-caseinate NP hydrogel as a nanocarrier. To improve enzyme retention and preserve their activity. To create a suitable substance for 3D printing and enhance the mechanical properties of the scaffold, cellulase-functionalized chitosan hydrogel was reinforced by CNFs. Cell survival and proliferation were enhanced by cellulase, which caused regulated biodegradation of the cellulose. CNFs can be generally produced by the disintegration of wood pulp [150]. However, it needs more than 25000 kWh/ton of energy, making this process unfavorable [151].

Consequently, enzymatic treatments can be beneficial before or after homogenization to reduce energy consumption. Cellulase has been widely used for the hydrolysis of cellulose to make CNFs in their free form [152,153]. However, using cellulase in the free state is proper for only one-time use since separating it from the reaction blend is difficult. It can be used several times without remarkably altering the performance of the enzyme, with lower energy consumption will be reduced. Moreover, it has also been demonstrated that immobilizing cellulase increases enzyme functioning stability due to increased resistance to reaction conditions such as temperature and pH [154].

Proteases (peptidases or proteolytic enzymes) can catalyze the cleavage of peptide bonds in proteins. It was classified into different categories based on its chemical structures and functional sites. Proteases come in wide different varieties, including serine-, metallo-, carboxyl-, acidic-, neutral-, and alkaline proteases. Bacteria and fungi account for most protease sources but can also be derived from animal tissues and plants [155]. Protease has been used in several industries, including textile, leather, pharmaceutical, and waste recycling [156]. Several investigations have been done to understand protease's different aspects and advantages. For instance, physical adsorption was used to immobilize protease on the untreated and NaOH-treated cellulose monoacetate/chitosan nanofibers. A morphological analysis shows that following an enzyme activity test, the uniform nanofiber shape changes to a more interpenetrated and flattened structure. The greatest immobilization yield obtained for glutaraldehyde-treated cellulose monoacetate/chitosan samples is around 83 %. In a study, PVA/chitosan nanofibers were surface-modified by immobilizing the keratinolytic proteases to deal with the problem of degradation of feathers from poultry industries. The 88 % efficiency was reported due to the immobilization of the keratinolytic proteases on PVA/chitosan nanofibers [157].

There are various advantages for bio surface modification that have made them an ideal selection to be preferred to physical and chemical surface modification. Using enzymes for bio-surface modification can help reduce toxic, hazardous chemicals such as metal catalysts, acids, and bases while modifying nanofibrous materials. Also, the process of enzymatic treatments is short and needs less energy, which leads to lower production of CO_2_ and water consumption. Therefore, modifying processes can save time and increase the efficiency of modifying procedures. On the other side, there are some limitations while utilizing bio-surface treatments. For instance, the high cost of enzymes, the lower reaction rate, and restrictions on operation conditions, as some enzymes are sensitive to pH and temperature that may restrict their usage. Future studies should consider the optimum conditions and applications to substitute enzyme treatment with classical techniques of surface modifications.

## 5 Application of modified nanofibrous material

### 5.1 Electrospun nanofibrous scaffolds for tissue engineering applications

Nanofibers present considerable benefits in tissue engineering because they can closely replicate the extracellular matrix (ECM), which aids in cell adhesion, proliferation, and differentiation. Their high porosity and inter-connectivity promote effective nutrient and waste exchange, essential for the survival of cells and the growth of tissue. Moreover, nanofibers can be tailored to have specific mechanical properties that align with those of the intended tissue, providing necessary support and flexibility. They can also be modified with bio-active molecules, growth factors, and drugs to encourage particular cellular responses and boost tissue regeneration. The diverse fabrication techniques, such as electrospinning, enable the creation of nanofibers from a variety of natural and synthetic polymers, allowing for the customization of nanofiber characteristics for different tissue engineering uses. These properties render nanofibers a highly promising material for the advancement of sophisticated tissue engineering scaffolds [158,159].

Nanofibrous materials have been widely used for many biomedical applications (Fig. 9).

**Fig. 9:** Applications of nanofibrous materials.

Surface modification of nanofibers is essential in tissue engineering and improves the interaction between nanofibers and biological tissues, which is vital for effective cell adhesion, proliferation, and differentiation. Recent research has indicated that modifying surfaces can greatly enhance the bio-compatibility of nanofiber scaffolds. For instance, PLLA nanofibers underwent surface modification through oxygen plasma treatment to add hydroxyl functional groups. Subsequently, cationic gelatin was chemically grafted to the modified nanofibers. The findings indicated improved viability, proliferation, and differentiation of rabbit articular chondrocytes when compared to the unmodified PLLA nanofibers [160]. Also, the surface of PCL nanofibers underwent physicochemical modifications by subjecting to simultaneous soft X-ray/extreme ultraviolet (SXR/EUV) radiation and low-temperature nitrogen and oxygen plasma induced by SXR/EUV. The physical and chemical modifications on the treated PCL nanofiber surface were analyzed using SEM and X-ray photoelectron spectroscopy. It was reported that the scaffolds exposed to ionizing radiation and low-temperature plasma experienced significant chemical modifications, including the formation of several new chemical groups. Additionally, a smoothing effect on the PCL nanofiber surfaces was noted, characterized by the reduction or near-elimination of micropore size on the nanofibers. Furthermore, an increase in the viability and adhesion of 7F2 osteoblasts on the modified PCL nanofibers was demonstrated after 24 h of cell culture. These results showed that the surface-modified PCL nanofibers can be a promising candidate for tissue engineering [161]. A study focused on surface-modified nanofibers for bone tissue engineering as a nanofibrous scaffold composed of PCL, gelatin, and chitosan (PCL-GT-CS) was initially made using electrospinning techniques. The produced scaffold underwent treatment with 1 wt% nanohydroxyapatite (nHAp) for 10-, 20-, and 30-min. Results showed the uniform surface modification of nanofibers led to higher cell viability, effective cell attachment, and significant cell proliferation. Therefore, surface-modified nanofibers were suggested as efficient scaffolds for bone tissue engineering [162].

Table 6 illustrates different applications of various nanofibers in tissue engineering.

**Table 6:** Different applications of different nanofibers, their advantages, and methods of electrospinning.

Nanofiber(s)	Electrospinning type	Brief function or advantages	Application target	Ref
PC/chitosan	Needle	• Superior mechanical properties • Improved cell adhesion and proliferation of Schwann cells	Neural tissue engineering	[163]
PLGA	Coaxial	• Significant nerve regeneration	Sciatic nerve	[164]
Silk fibroin/P(LLA/CL)	Coaxial	• Sustained release of growth factor • Bioactivity for a long time • Promoted peripheral nerve regeneration	Sciatic nerve	[165]
PC/keratin	Needle	• Good blood compatibility • Better cell adhesion and proliferation than pristine PCL • Good cytocompatibility and blood compatibility	Vascular tissue engineering	[166]
Silk fibroin/poly(lactide-co-caprolactone)	Needle	• Improved mechanical properties, surface roughness, bone regeneration, and wettability • Better cell adhesion and proliferation • Robust osteogenic differentiation capability	Bone tissue regeneration	[167]
PCL/chitosan/gelatin	Needle	• Enhanced cell adhesion and viability • Good mechanical properties • An appropriate rate of water vapor transmission • Remarkable swelling	Skin tissue scaffolds	[168]

In summary, nanofibers offer significant advantages in tissue engineering due to their high surface area, porosity, and ability to mimic the extracellular matrix (ECM). They enhance cell adhesion, proliferation, and differentiation, making them ideal scaffolds for tissue regeneration. However, challenges include ensuring uniform fiber distribution and mechanical strength, as well as potential issues with biocompatibility and degradation rates. Future research should focus on optimizing fabrication techniques and improving the functional properties of nanofibers to overcome these challenges.

### 5.2 Electrospun nanofibers as bio masks (particularly for COVID-19 prevention)

Since the first case of COVID-19 was reported in December 2019, researchers have been working tirelessly to understand the origin, clinical signs, and transmission of the disease, as well as developing prevention methods and vaccines. As a result of this pandemic, bio masks have become a crucial component of daily life for individuals worldwide, with a particular emphasis on their use in preventing the spread of the virus [[169], [170], [171], [172], [173], [174], [175]]. These masks are designed to protect the wearer from airborne particles, including infectious agents like the SARS-CoV-2 virus. Electrospun nanofibers have been investigated as a potential material for bio masks due to their high surface area-to-volume ratio, allowing for efficient particle filtration. However, the properties of electrospun nanofibers can be further enhanced through surface modification. Surface modification can improve bio mask filtration efficiency, breathability, and antiviral properties.

One common approach to surface modification of electrospun nanofibers is using NPs. NPs can be incorporated into the electrospinning process, forming composite nanofibers with enhanced properties. For example, silver NPs have been widely used for surface modification of electrospun nanofibers due to their excellent antimicrobial properties [176]. Tebyetekerwa et al. [177] discussed the mechanisms and uniqueness of electrospun nanofibers in facemasks, along with DIY steps for creating functional facemasks at home. They also addressed the challenges and opportunities of nanofiber-based facemasks, including surface modification techniques such as hydrophobic polymer coatings and incorporating natural extracts or essential oils. Furthermore, they mentioned some standards such as, MIL-M-36954 C: ΔP, ASTM F1862, ASTM F2299, and ASTM F2101 for determining different physical properties of the face masks. They showed that porosity of electrospun layers, breathability and efficiency can be controlled by altering the parameters of electrospinning. Naragund and Panda [178] provided an overview of recent developments in electrospun nanofiber-based respiratory face masks, covering materials, fabrication techniques, performance parameters, and testing standards. They also discussed surface modification methods such as PU or PVA coatings and GO or ZnO NP functionalization. In another study, Essa et al. [179] reviewed different types of face masks and respirators, their filtration mechanisms, and their advantages and disadvantages. They also highlighted the role of nanofiber-based face masks and respirators in COVID-19 protection and discussed surface modification methods such as chitosan or gelatin coatings and silver or copper NP functionalization, among others. Sana Ullah et al. [180] compared melt-blown (MB) filters, commonly utilized in N95 face masks, with nanofiber filters gaining recognition as highly effective for mask filtration, to evaluate their reusability. Two modification methods were implemented: in the first, samples were immersed in 75 % ethanol, while in the second, 75 % ethanol was sprayed onto the samples. The findings revealed that the filtration efficiency of the MB filter significantly decreased following treatment with ethanol, whereas the nanofiber filter consistently maintained high filtration efficiency regardless of the cleaning method used. Furthermore, the nanofiber filter displayed superior cytocompatibility in comparison to the MB filter, indicating its safety for human use. Both filter types retained their hydrophobic surfaces despite the ethanol treatments, effectively preventing wetting from moisture and saliva splashes, thereby inhibiting pathogen transmission and bacterial growth.

Nikhil Avinash Patil et al. [181] developed a biodegradable face mask with a 3-ply structure made of cotton-PLA-cotton, featuring encapsulated phytochemicals in the inner filtration layer. The nano-fibrous PLA filtration layer was created through needleless electrospinning using PLA combined with herbal extract-based phytochemicals. This three-layer face mask demonstrates improved air permeability, showing a differential pressure of 35.78 Pa/cm^2^, and boasts an outstanding bacterial filtration efficiency of 97.9 % compared to commercial face masks. The filtration layer was able to effectively capture particulate matter, aerosol particles, and bacterial elements because of the densely packed mesh configuration of the nano-fibrous mat. The outer hydrophobic layer of the mask showed effective resistance to blood splashes up to a distance of 30 cm, which makes it suitable for medical applications.

In conclusion, nanofibers are advantageous in drug delivery systems due to their high porosity, large surface area, and ability to control drug release kinetics. They enable targeted and controlled drug delivery, enhancing therapeutic efficacy and reducing side effects. However, challenges including uniform drug loading and release, and the stability of the nanofibers should be the aims of future investigations to develop stimuli-responsive nanofibers and improve the biocompatibility and stability of these systems.

### 5.3 Electrospun nanofibers for drug delivery systems

The fundamental purpose of using advanced biomaterials as drug delivery systems is to administer a specified quantity of medicine at a specific rate. Nanofibrous membranes are strongly recommended as a delivery method because they offer promising characteristics such as a large surface area to volume ratio, which leads to regulated drug delivery. Site-specific delivery and bloodstream transport are the two main drug delivery systems. Many nanofibrous membranes can only transport medications to different tissues [182]. The ability of electrospun nanofibers in drug delivery depends on their particular activity and intrinsic nanoscale structural properties [183].

Furthermore, because of the conventional manufacturing flexibility, several structural topologies, including therapeutic molecules, might be created from monolithic nanofibers for diverse applications [184]. These advantages enable finely controlled drug-solubilized profiles based on adjusting drug traveling length or changing the attraction between matrix materials and pharmaceuticals. The mechanism of drug release is linked to polymer breakdown and a complicated diffusion way via nano-scaled void spaces inside nanofiber mats. Various formulation factors, such as polymer characteristics, polymer type, surface coating, and drug molecule state in a solid phase, effectively modify drug release patterns [185]. The fibrous surface structure appears solid adhesiveness to mucous layers since their nano-porous forms immediately assimilate dampness at mucous layers through nano-void volumes. The prevalent adhesiveness toward natural surfaces makes nanofibers a perfect candidate for topical medicate conveyance gadgets [186]. In a study, chitosan and alginate were deposited on PLGA nanofibers to form a multilayer by the LBL assembly. Surface functionalization made the surface positive, confirmed by the potential zeta test, and led to regular interactions between the LBL coating and loaded ibuprofen. The nanofibers were pH-sensitive due to variations of drug release in acidic pH (1.0), and neutral pH made them a successful candidate for drug delivery systems [187]. Namita Ojah et al. [188] showed that dielectric barrier discharge (DBD) oxygen (O_2_) plasma modifies electrospun Bombyxmori silk/Amoxicillin hydrochloride trihydrate (AMOX)/PVA nanofibers for drug release applications, varying the plasma treatment time from 1 to 10 min. The electrospun nanofibers treated for 1–3 min experienced a significant improvement in surface energy, Young's modulus, tensile strength, and wettability. Nanofibers exposed to plasma treatment for 1–5 min demonstrated a notable increase in the rate of AMOX release, while those treated for longer than 5 min indicated only slight enhancement. Additionally, the plasma-treated nanofibers exhibited effective antibacterial activity against both *E. coli* and *S. aureus* bacteria. In another study, the composite membranes of zeolitic imidazolate framework-8 and polylactic acid (ZIF-8/PLA) were created using a secondary growth technique on the surface of an electrospun nanofiber membrane. As the incubation time increased and the concentration of 2-methylimidazole (2-MIM) rose, the size of the ZIF-8 particles became larger and uniformly distributed on the surface of nanofibers led to enhanced hydrophilicity and surface roughness. Additionally, the PLA/ZIF-8 nanofiber membranes demonstrated remarkable pH sensitivity and drug release capability. Whereas only about 40 % of the encapsulated drug was released in a buffer with a pH of 7.4, more than 90 % was released at a pH of 5.5 due to the dissolution of the ZIF-8 framework in acidic solutions [189].

Nanofibers enable targeted and controlled drug delivery, enhancing therapeutic efficacy and reducing side effects. However, challenges include ensuring uniform drug loading and release, stability of the nanofibers in the in vivo applications, and biocompatibility should be focused on in future studies.

### 5.4 Electrospun nanofibers in biomembranes

The electrospun nanofibers are widely used in biomembranes with various applications such as tissue engineering and drug delivery systems [190,191]. A wide range of synthetic and natural polymers have been used such as poly (vinyl chloride) (PVC), PLLA, polystyrene (PS), alginate, silk fibroin, chitosan, and chitin [192]. Research showed that any variation in electrospinning parameters changes the morphology of the nanofibers, improving the drug loading and releasing and mechanical properties of the membranes [192,193]. Dimethyloxalylglycine (DMOG)-loaded mesoporous silica NPs and PLA were used to prepare nanofibrous membranes for wound healing application. Appropriate drug delivery and a higher rate of diabetic wound healing were the results of well-shaped nanofibers [194]. The co-electrospinning process is used to develop a PCL/gelatine-based membrane. Adjusting the PCL nanofibers resulted in a controlled drug release profile and degradation rate of gelatin [195]. The LbL method was used to form chitosan and alginate layers on PLGA nanofibers to create a pH-sensitive membrane, controlling ibuprofen release in an acidic stomach and optimizing release at higher pH [196]. Tyubaeva et al. [197] produced a nanofibrous membrane that surfaces modified with poly-3-hydroxybutyrate (PHB) and natural environmentally friendly additives of iron-containing porphyrin and Hemin (Hmi). Evaluations of the resulting membranes showed an improvement in wettability and surface morphology. In addition, the produced bio-compatible membranes showed remarkable air and liquid permeability.

Biomembranes from nanofibers offer high mechanical strength, biocompatibility, and tunable surface properties, making them suitable for various medical applications, including filtration and tissue regeneration. However, limitations such as uniform fiber distribution and maintaining the structural integrity of the membranes should be investigated. Current issues involve the scalability of production and the cost of materials. Therefore, developing cost-effective and scalable fabrication methods can enhance the functional properties of nanofibrous biomembranes in the lab and industrial scales.

### 5.5 Electrospun nanofibers in wound dressing

Chronic wounds are issues that patients with diabetes and burns suffer. Appropriate treatments cost up to €2–2.5 billion in Europe [198] and more than $25 billion annually in the USA [199]. Diverse methods and nanofibrous materials were used in wound dressing. For instance, electrospun core-shell nanofibers of amoxicillin trihydrate-silk (core)/PVA (shell) were produced as a drug delivery system and functional wound dressing. Core-shell nanofibers were then surface-modified by plasma treatment. Surface modification of nanofibers introduced hydrogen bonds on the surface, leading to higher mechanical properties. Moreover, biological tests proved the application of modified nanofibers in wound dressing [200]. Yang Jun et al. [201] developed MOF-coated PAN/gelatin nanofibers to control drug release and wound healing. Surface modification of nanofibers using MOF and gelatin improved the antibacterial activity and drug loading capacity, leading to five days of shorter wound healing. PVA nanofibers based on hyaluronic acid (HA) were used as an effective ECM. L-arginine was loaded on citric acid and then cross-linked to the PVA-HA nanofibers. These nanofibers showed low mechanical properties, which were then modified by cellulose nanocrystals (CNCs). Surface-modified nanofibers were examined by melanocyte (HFB-4) and lung fibroblast (WI38) cells. Results confirmed the high efficiency of modified nanofibers in skin wound healing applications [202]. The research conducted by Kalaoglu-Altan et al. [203] investigated the use of electrospun fibers from silver nanoparticle-coated polyhydroxyalkanoate (PHA) in wound dressings, emphasizing several important surface modifications to promote wound healing. Silver nanoparticles provide potent antimicrobial effects, significantly lowering the risk of infections and keeping the wound environment cleaner. The biocompatibility and biodegradability of PHA facilitate cell attachment and growth, which are essential for tissue regeneration. Furthermore, the electrospun fibers can be designed for the controlled release of drugs, allowing for the continuous delivery of therapeutic agents directly to the wound site. This mechanism of controlled release is crucial for maintaining effective drug levels over prolonged periods. The structure of the nanofibers is also important for moisture management, assisting in maintaining an optimal moisture balance for quicker wound healing and minimizing scarring. Together, these surface modifications foster a protective, antimicrobial, and nurturing environment for effective tissue repair, highlighting the potential of these innovative materials to enhance wound care results. In another study, cyanoethyl chitosan electrospun nanofibers were used to assess the healing performance of wound dressing. Electrospinning parameters such as solution concentration, field, and feed rate were changed and various samples were prepared. Antibacterial assessments showed the highest contact kills at 8–10 % of solution concentration against different bacteria. Moreover, finer fibers showed higher surface area leading to better antibacterial performance [204].

Nanofibrous wound dressings provide a moist healing environment, promote cell proliferation, and can be functionalized with antimicrobial agents and growth factors. They offer advantages such as high porosity, facilitating gas exchange, and exudate management. Primary challenges such as consistent production quality and maintaining the mechanical strength of the dressings can be the goals of future investigations. Current issues involve the cost of production and the need for more effective antimicrobial agents. Ongoing research is trying to optimize the composition and functionalization of nanofibrous wound dressings to improve their therapeutic potential.

### 5.6 Electrospun nanofibers in biosensors

The necessity for analytical instruments to identify and monitor specific analyses has grown as numerous needs for medical diagnostics and environmental protection. Sensors and biosensors allow to sensing of various materials in gas sensing. Nanofibers and films of cellulose acetate-glycerol-conducting polymer-WO_3_ NPs were produced by Rahman et al. as H_2_S gas sensors. The developed sensors performed admirably at room temperature (20 °C). These sensors could detect a gas concentration of 1 ppm and show stability and repeatability without affecting the humidity [205]. In a similar study, WO_3_ nanofibers, sensitive to NO_2_, were produced through electrospinning with the morphology and particle size dependent on the heating rate. In addition, the interaction between the surface of the nanofibers and NO_2_ was the leading of the high selectivity against low and high concentrations of NO_2_ [206]. Nanofiber-based sensors could also be used as human health and body movement monitors [207]. Abolhasani et al. [208] developed graphene/PVDF porous nanofibers to sense movement. Results showed that 0.1%wt graphene could increase the voltage response to 14.8 ± 2.1 V, three-fold more than the pristine PVDF nanofibers.

Nanofibrous structures are ideal for biosensors due to their high surface area, conductivity, and ability to immobilize biomolecules. They enable the development of sensitive and selective diagnostic tools for detecting various analytes. Drawbacks include the stability and reproducibility of the sensors, as well as the potential scalability of production that may limit the use of nanofibers in this field. Therefore, improving the stability and scalability of nanofiber-based biosensors and developing new applications for these diagnostic tools may be the solution to overcome these restrictions.

## Summary and outlook

Nanofibrous materials have garnered significant attention for their potential in diverse applications, particularly within the medical field. This review has explored various surface modification techniques that enhance the functionality of nanofibers, such as electrospraying plasma treatment, and chemical vapor deposition. These techniques have been instrumental in tailoring the surface properties of nanofibers to meet specific biomedical needs. For instance, the bioactive molecules and antimicrobial agents has shown promising results in wound healing and tissue engineering applications. Despite these advancements, certain limitations persist. Hydrophobicity can impede cell adhesion and proliferation on nanofibrous scaffolds, which is critical for tissue engineering applications where hydrophilic surfaces are often required to support cell growth and differentiation. Addressing these limitations through innovative surface modification strategies is essential for the continued progress of nanofibrous textiles in biomedical applications. Several key areas warrant further research to realize the potential of nanofibers in medical applications. First, developing multifunctional nanofibers that simultaneously address multiple biomedical challenges, such as infection control and tissue regeneration, is a promising direction. This could involve the integration of various bioactive compounds and smart materials that respond to environmental stimuli. Additionally, exploring eco-friendly and sustainable surface modification techniques will be crucial. As the demand for green technologies grows, finding ways to modify nanofibers without relying on harsh chemicals or energy-intensive processes will become increasingly important. Finally, more in-depth studies on the biocompatibility and biodegradability of modified nanofibers are needed. Understanding how these materials interact with biological systems over extended periods will help in safer and more effective medical devices and implants. By addressing these areas, future research can pave the way for the next generation of nanofibrous materials that are not only highly functional but also sustainable and biocompatible.

## CRediT authorship contribution statement

**Rasool Shabanloo:** Writing – original draft, Investigation. **Majid Montazer:** Writing – review & editing, Validation, Supervision, Conceptualization. **Ali Farahani:** Writing – original draft, Investigation. **Nesa Karimi:** Writing – original draft, Investigation.

## Declaration of competing interest

The authors declare that they have no known competing financial interests or personal relationships that could have appeared to influence the work reported in this paper.

## Data Availability

No new data was generated for the research described in the article.
